# Increased Six1 expression in macrophages promotes hepatocellular carcinoma growth and invasion by regulating MMP‐9

**DOI:** 10.1111/jcmm.14342

**Published:** 2019-05-02

**Authors:** Yongyu Zhang, Shiji Wang, Zhongmin Liu, Lewei Yang, Jian Liu, Ming Xiu

**Affiliations:** ^1^ Department of Interventional Radiology The Fifth Affiliated Hospital of Sun Yat‐sen University Zhuhai China; ^2^ Department of Intensive Care Unit The First Hospital of Jilin University Changchun Jilin China; ^3^ Department of Radiation Oncology The Fifth Affiliated Hospital of Sun Yat‐sen University Zhuhai China; ^4^ Department of Infectious Diseases The Fifth Affiliated Hospital of Sun Yat‐sen University Zhuhai China

**Keywords:** hepatocellular carcinoma, invasion, MMP‐9, Six1, STAT3

## Abstract

Increased Six1 expression is commonly observed in a variety of cancers and is positively correlated with cancer progression and metastasis. Nevertheless, the mechanism by which Six1 affects the development of hepatocellular carcinoma (HCC) is still unclear. A series of experiments involving cell counting kit‐8, colony formation and Transwell assay was used to determine cell proliferation, migration and invasion respectively. Histological examination and immunofluorescence assay were also performed. The messenger RNA and protein expression of interesting genes were determined by real‐time reverse transcription‐polymerase chain reaction and western blotting respectively. We found that Six1 was up‐regulated in HCC and was associated with worse histological grade and poor survival rate. Increased expression of Six1 was shown to be able to boost cell growth, invasion, migration and epithelial‐mesenchymal transition (EMT), whereas silencing of Six1 suppressed these malignant phenotypes. Mechanistic investigations revealed that, in macrophages, matrix metalloproteinase 9 (MMP‐9) was up‐regulated by Six1. Interestingly, Six1 expression in macrophages was also able to trigger MMP‐9 induction in HCC cells. Moreover, macrophage Six1 expression was able to induce interleukin‐6 (IL‐6) up‐regulation and increase the activity of signal transducer and activator of transcription 3 (STAT3) in HCC cells, which accounted for the elevated levels of MMP‐9 and the higher invasive levels seen in HCC. Increased expression of Six1 in HCC aggravates the malignant behaviour of cancer cells, and we provide novel evidence that macrophage Six1 can stimulate cancer cell invasion by elevating MMP‐9 expression.

## 1 INTRODUCTION

Hepatocellular carcinoma (HCC) ranks fifth as one of the world's most common cancers.^1^, ^2^ Although the survival rate for HCC patients has increased owing to improvements in treatments as well as scientific advances in understanding the aetiology of HCC, post‐surgery survival rates after resection remain relatively low, with metastasis being the main reason for the low survival rate.^3^, ^4^ Despite this, the mechanisms underlying the ability of HCC to metastasize and invade other tissues remain obscure. Therefore, understanding of these underlying mechanisms remains an important goal in HCC treatment.

Tumour‐associated macrophages (TAMs), the numerous immunocytes found in the tumour cell microenvironment, are regarded as being important in HCC metastasis and invasion.^5^, ^6^ It has been demonstrated that a significant elevation in TAM infiltration is often connected with higher mortality, which suggests that TAMs can facilitate tumour development.^7^ Macrophages are critical for tumour metastasis through the production of matrix‐metalloprotease 9 (MMP‐9).^8^, ^9^ The action of MMP‐9 may undermine the basilar membrane and extracellular matrix (ECM), thus fostering a beneficial environment for cancer progression.^10^, ^11^ Owing to the significant role played by TAMs in tumour progression, an increasing number of treatment strategies have been formulated to target major molecules in macrophages.^12^ Recently, several molecules have been found to be expressed in macrophages that play crucial roles in tumour pathogenesis.^13^ Genetic research in mice has shown that the absence of the epidermal growth factor receptor (EGFR) in liver macrophages hinders the development of HCC, whereas the absence of EGFR in hepatic cells improves their ability to proliferate, thus facilitating the progression of HCC.^1^, ^14^ This is thought to be the principal reason that therapeutic strategies that target the EGFR might not be of use in late‐stage HCC patients.^1^ Eliminating the receptor for advanced glycation end products in macrophages has also been shown to prolong the lives of mice with glioma because of improved angiogenesis and a decline in TAM‐related inflammation and angiogenesis.^15^ Based on this, further study is needed to investigate the underlying molecular mechanisms by which macrophages influence cancer progression.

As a homoeodomain protein in the Six family, Six1 plays a crucial role in organ growth.^16^ Its high expression has been found in multiple cancers and is closely correlated with aggressive cancer as well as increased mortality.^16^, ^17^ Higher levels of Six1 expression are also associated with lower overall survival rates in late‐stage (III & IV) CRC patients, in whom metastasis was shown to have extended to certain lymph nodes.^18^ In addition, overexpression of Six1 is also found in non‐metastatic early to middle‐stage (I‐III) CRC patients, correlating with an unfavourable prognosis in both groups.^19^ Experiments using an RNA intervention approach have shown that there is a suppressive effect of lower Six1 expression on cancer progression and invasion.^20^

In the current study, we show that Six1 is more highly expressed in macrophages compared to that in adjoining healthy tissues in HCC patients. We also demonstrate that overexpressing Six1 in macrophages stimulates cancer cell invasiveness. Six1 overexpression can increase the levels of the matrix metalloprotease MMP‐9 through the NF‐κB/p65 signalling pathway in macrophage. Moreover, Six1 expression in macrophages triggers the IL‐6/STAT3/MMP‐9 pathway, subsequently facilitating tumour cell invasion. Our study indicates that Six1 expression not only increases MMP‐9 expression in macrophages but also increases MMP‐9 expression in tumor cells. Our data therefore offer new thoughts on the role of Six1 in HCC invasion, providing a basis for formulating therapeutic strategies that could target Six1 expression in macrophages, as a future goal.

## 2 MATERIALS AND METHODS

### 2.1 Cell culture

Cancer cell lines THP‐1, HA59T and HepG2 were obtained from American Type Culture Collection (ATCC). The HA59T and HepG2 cells were cultured in DMEM medium containing 10% foetal bovine serum (FBS). Human THP‐1 cells were cultured in RPMI1640 medium. To differentiate to macrophage, THP‐1 cells were cultured with PMA (15 ng/mL), using dimethyl sulphoxide as the vehicle, for 24 hours.

### 2.2 Tissue microarrays and immunohistochemical staining

Two paraffin‐embedded HCC tissue arrays, with associated patient survival information, were purchased from SuperBioChips Laboratories. These microarrays were cultured with a 1:200 dilution of an anti‐Six1 antibody. Immunological staining was performed using 3,3‐diaminobenzidine (Sigma). The distribution and positive signal intensity of Six1 staining were graded by two independent graders, with the grading principle set upon the proportion of positive tumour cells in tissues (0, 0%; 1, <25%; 2, 25%‐50%; 3, 51%‐75%; and 4, >75%) as well as the intensity of staining. The staining scores over 6 were considered being representative of high expression levels. The patients or their families provided signed informed consent.

### 2.3 Cell viability and colony formation

HA59T or HepG2 cells (5 × 10^4^) were seeded into six‐well plates together with culture medium. Viable cells were examined using the trypan blue dye exclusion assay at time points of 0, 24, 48 and 72 hours. For the anchorage‐dependent cell colony formation assay, cells were put in six‐well plates (500/well) and incubated for 14 days. Colonies were fixed and then stained with gentian violet prior to counting.

### 2.4 Cell invasion and migration assay

Transwell inserts in 24‐well plates containing uncoated filters (8 μm in pore size) were used to assess cell migration and Matrigel (BD Biosciences)‐coated filters were used to assess cell invasion. Cells (2 × 10^4^) in 0.2 mL serum‐free DMEM were put into the inserts, and 0.6 mL of DMEM medium was placed in the lower section of the well. HA59T and HepG2 cells were incubated for 48 hours. Three independent experiments were performed in total.

### 2.5 Histological examination

Formalin fixed and paraffin embedded HCC tissue sections were obtained from the Department of Intensive Care Unit, First Hospital of Jilin University. Epidermoid carcinoma was diagnosed by either cytological or pathological evidence. Sections of non‐tumour and tumour tissues were cut to a thickness of 5 μm. Serial tissue sections were deparaffinized and rehydrated; then, antigen retrieval was carried out. Nearby non‐tumour tissues were isolated at room temperature for 10 minutes to prevent binding before incubation with the rabbit anti‐Six1 antibody, the mouse anti‐CD68 (cluster of differentiation 68) antibody or the anti‐MMP‐9 antibody. The secondary antibodies used were goat polyclonal anti‐rabbit or anti‐mouse antibodies. HRP activity was detected using the chromogen substrate 3, 3′‐diaminobenzidine.

### 2.6 Transfection with siRNAs & plasmids

The PCMV‐XL4 Six1 plasmid was obtained from Addgene, and siRNAs targeting Six1(GCCAGGAGCUCAAACUAUU) and p65 (GGAGUACCCUGAAGCUAUAUU) were synthesized. THP‐1 cells were transfected with either the PCMV‐XL4 Six1 plasmid or siRNAs using Lipofectamine 2000 (Invitrogen, Carlsbad, CA, USA) according to the manufacturer's instructions.

### 2.7 Immunofluorescence assay

THP‐1 cells were pelleted and resuspended in medium (100 μL), and cells were fixed. THP‐1 cells were embedded in paraformaldehyde (4%) and then permeabilized for 10 minutes. THP‐1 cells were incubated with the appropriate antibodies overnight. Immunofluorescent staining was performed using anti‐Six1 and anti‐CD68 antibodies (Cell signaling Technology, MA, USA).

### 2.8 Cell counting kit‐8 (CCK‐8) analysis

CCK‐8 assay was used to detect cell viability. HA59T cells cultured in 96 wells for 24 hours with medium altered for the collection of CM. CCK‐8 analysis was then conducted 24, 48 and 72 hours after this. For analysis, CCK‐8 (10 µL) was added and the absorbance at 450 nm was detected using a BioTek.

### 2.9 Real‐time reverse transcription‐polymerase chain reaction (RT‐PCR)

RNA was harvested by TRIzol reagent and reverse transcription was performed using a First Strand cDNA synthesis Kit (Sigma). Real‐time RT‐PCR analysis was performed using Promega's GoTaq^®^ qPCR Master Mix. The following thermocycling conditions were used for the real‐time RT‐PCR: Initial denaturation at 94°C for 1 minute; 35 cycles for 94°C for 1 minute, 60°C for 1 minute, 72°C for 1 minute; and a terminal extension at 72°C for 5 minutes. Quantitative determination of messenger RNA (mRNA) levels was performed using β‐actin for normalization. The following primer sequences were used to detect the level of the relevant human mRNAs: β‐actin: F: 5′‐CCAACCGCGAGAAGATGA‐3′, R: 5′‐CCAGAGGCGTACAGGGATAG‐3′; Six1: F: 5′‐TTACGCAGGAGCAAGTGGCG‐3′, R: 5′‐CGCTCTCGTTCTTGTGCAGG‐3′; MMP‐9: F: 5′‐TTGACAGCGACAAGAAGTGG‐3′, R: 5′‐GCCATTCACGTCGTCCTTAT‐3′; IL‐6: F: 5′‐AAGCCAGAGCTGTGCAGATGA GTA‐3′, R: 5′‐TGTCCTGCAGCCACTGGTTC‐3′.

### 2.10 Western blotting

Total protein lysate was harvested as previously described.^21^ Protein concentration was determined by Piece BCA protein Assay kit (Thermo Fisher Scientific) and was separated by 10% SDS‐PAGE and transblotted onto polyvinylidene difluoride membranes (PVDF). Next, PVDF membranes were blocked using 5% not‐fat milk in tris‐buffered saline for 1 hour at room temperature, and membranes were incubated with primary antibodies at 4°C overnight. After washed, the membranes were incubated with the appropriate secondary antibodies for 1 hour at room temperature. Finally, an enhanced chemiluminescence ECL Detection Kit was used to evaluate the bands, and a transilluminator was used to examine the intensity of the image. The primary antibodies included anti‐Six1, anti‐MMP‐9, anti‐p‐STAT3, anti‐STAT3, anti‐p65 and anti‐β‐actin (Cell signaling Technology, MA, USA).

### 2.11 Statistical analysis

All statistic evaluation was performed using GraphPad Prism V. A Student's *t* test was applied for analysis. A two‐sided Fisher test was used to compare Six1 expression with clinical and pathological characteristics. A Kaplan‐Meier assay and a log‐rank test were also conducted to gauge overall survivability. *P* < 0.05 was considered statistically significant.

## 3 RESULTS

### 3.1 Six1 expression is up‐regulated in HCC and relative to poor progression

The protein expression of Six1 in HCC was examined using tissue microarrays taken from different patients. Six1 expression level was high in tissues from patients with invasive HCC, compared to those in tissues from patients with non‐invasive HCC, or patients with benign tissue samples (Figure 1A and B). HCC patients with disease recurrence had higher levels of Six1 mRNA expression than patients who did not experience recurrence (Figure 1C). Additionally, for patients with and without metastases, the Six1 mRNA level was considerably higher in HCC tissues of the former compared to those of the latter (Figure 1D). We also found that a much lower survival rate in HCC patients with high level (n = 56) of Six1 compared to that in patients with low Six1 level (n = 57; Figure 1E). These data show that there is a consistent up‐regulation of Six1 in HCC, and that its expression is positively correlated with high histology grade and poor prognosis.

**Figure 1:** Six1 overexpression relates to poor prognosis and promotes hepatocellular carcinoma (HCC) metastases. A, Representative images of immunohistochemical (IHC) staining of Six1 protein in HCC tissue microarrays. B, Six1 staining IHC scores in benign breast disease (n = 5), non‐invasive HCC (n = 6), and invasive HCC tissues (n = 6). C, Relative mRNA expression of Six1 in HCC samples from patients with disease recurrence (n = 20) or without disease recurrence (n = 20). D, Relative mRNA expression of Six1 in HCC samples from patients with metastasis (n = 17) or without metastasis (n = 18). (E) Kaplan‐Meier analysis for patients with HCC. The analyses were conducted based on the immunohistochemical score for Six1 and the survival information provided by the supplier of the HCC tissue microarray. Log‐rank test, n = 113, *P* = 0.008. Data are presented as means ± SD. *P < 0.05; **P < 0.01; ***P < 0.001

### 3.2 Six1 regulates the malignant phenotype and EMT in HCC cells

To explore the impact of Six1 on malignant characteristics in HCC cells, cell growth, colony formation, invasion and metastases were examined. We found that overexpression of Six1 boosted cell growth, whereas knockdown of Six1 mildly decreased cell growth (Figure 2A). Consistently, overexpression of Six1 increased the number of anchorage‐dependent colonies, whereas knockdown of Six1 slightly decreased the number of colonies (Figure 2B). Interestingly, overexpression of Six1 dramatically promoted FBS‐induced invasion and metastases, whereas reduction of Six1 levels significantly hindered invasion and metastases (Figure 2C and D). As cell invasion and morphological changes are tightly associated with the EMT, we then evaluate the level of the epithelium markers, ZO‐1, E‐cadherin and mesenchymal marker vimentin by western blotting. The data showed that overexpression of Six1 suppressed the expression level of ZO‐1 and E‐cadherin, while increasing vimentin levels in HA59T cells. In contrast, knockdown of Six1 increased the expression level of ZO‐1 and E‐cadherin, but down‐regulated vimentin expression levels in HA59T cells (Figure 2E). These data indicate that Six1 can modulate HCC cell growth, colony formation, migration, invasion and the EMT in vitro.

**Figure 2:** Effect of Six1 expression on the malignant phenotype in hepatocellular carcinoma (HCC) cells. A, The cell viability of HA59T and HepG2 cells expressing different levels of Six1 were analysed at the indicated time points. B, The effect of different levels of Six1 expression on anchorage‐dependent colony formation. C, Six1 regulation of transwell cell migration and D, of Matrigel invasion. Overexpression of Six1 significantly enhances both migration and invasion in HA59T cells, whereas knockdown of Six1 suppresses migration and invasion in HepG2 cells at 48 h. Representative images are shown at the bottom. E, Expression of the epithelial markers, E‐cadherin and ZO‐1 and the mesenchymal marker, vimentin, were analysed by western blotting in the HA59T cells with or without Six overexpression and HepG2 cells with or without Six knockdown. Data are presented as means ± SD (n = 3). *P < 0.05; **P < 0.01

### 3.3 Six1 in macrophages stimulates the invasiveness in HA59T cells

Next, we conducted immunofluorescence staining for both Six1 and CD68 (a macrophage marker) in tumour and non‐tumour tissue samples.^22^, ^23^ Six1 was found to be higher expression level in macrophages HCC tissues than in non‐tumour tissues (Figure 3A).

**Figure 3:** Macrophage Six1 promotes HA59T cell invasion. A, Co‐immunofluorescent staining with Six1 and CD68 in cancer tissues and non‐tumour tissues. B, Representative images of THP‐1 cells treated, or not, with PMA. C, Real‐time RT‐PCR and western blotting analysis of Six1 expression in Six1‐MOE and Vector‐M cells (Upper). Real‐time RT‐PCR and western blotting analysis of Six1 expression levels in Six1‐MKD and Con‐MKD cells (Bottom). D, Cell viability of Six1‐MOE CM‐ or Vector‐M CM‐treated HA59T cells were evaluated by CCK‐8 assay. E, Cell viability of Six1‐KD CM or Con‐KD CM‐treated HA59T cells was evaluated by CCK‐8 assay. F, Quantitative analysis of HA59T cell invasion when co‐cultured with either Six1‐MOE or Vector‐M cells in the invasion assay. G, Quantitative analysis of HA59T cell invasion when co‐cultured with Six1‐MKD or Con‐MKD cells in the invasion assay. Data are shown as mean ± SD. **P < 0.01

THP‐1 cells were stimulated with PMA for 24 hours, after which cells were maintained in culture, morphological changes were clearly detected in the cells (Figure 3B). With the goal of understanding the role of macrophage Six1 in HA59T cell invasion, an invasion assay was conducted using macrophages having either increased or knocked down levels of Six1. Six1 expression in stimulated macrophages was determined by western blotting and real‐time RT‐PCR. Under normal conditions, Six1 expression could be observed in macrophages. The Six1 expression levels at both protein and mRNA were considerably higher in macrophages transfected with the pCMV‐XL4 Six1 (Six1‐MOE) plasmid than in cells transected with the control plasmid (Vector‐M; Figure 3C). It was also apparent that Six1 siRNA inhibited Six1 expression in macrophages (Six1‐MKD), compared to that in cells transfected with the control siRNA (Con‐MKD; Figure 3C).

A CCK‐8 assay was used to explore the impact of Six1 expression levels in macrophages on HA59T cell growth. Conditioned media (CM) was obtained from Six1‐MOE, Six1‐MKD, Vector‐M and Con‐MKD cells and used to treat HA59T cells. Culture of the HA59T cells with Six1‐MOE‐derived CM for 1 day, 2 days and 3 days failed to promote HA59T cell growth in contrast to that in cells administrated Vector‐M‐derived CM (Figure 3D). Culture in the presence of Six1‐MKD‐derived CM for same three time periods did not have effect on HA59T cell growth (Figure 3E).

As a result of these findings, we carried out a cell invasion assay for 1 day using Six1‐MOE and Six1‐MKD cells to investigate how Six1 expression in macrophages influences the invasiveness of HA59T cells to ignore the influence of cell viability. Based on our observations, the number of invading HA59T cells increased when they were cultured in the presence of Six1‐MOE cells vs Vector‐M cells (Figure 3F). Culture in the presence of macrophages with decreased Six1 levels (Six1‐MKD) drastically curbed the invasiveness of HA59T cells compared to that of Con‐MKD cells (Figure 3G). These findings indicate that Six1 has a critical role in facilitating HA59T cell invasion.

### 3.4 Impact of Six1 on MMP‐9 expression level

Macrophages are well known to be able to stimulate the invasion process and metastasis of cancer cells, partly through inducing the expression of MMP‐9 which leads to matrix remodeling.^1^ In order to fully explore the underlying mechanism by which Six1 expression in macrophages affects the invasiveness of HA59T cells, we examined MMP‐9 expression level in macrophages having different levels of Six1 expression. As shown in Figure 4A, there was increased MMP‐9 mRNA levels in Six1‐MOE cells compared to Vector‐M cells. In addition, Six1 siRNA considerably decreased the mRNA expression level of MMP‐9 in Six1‐MKD cells compared to Con‐MKD cells, as shown in Figure 4B. These observations were confirmed by western blotting for MMP‐9 in the various macrophage cell lines. A higher level of expression of MMP‐9 was found in Six1‐MOE cells compared to Vector‐M cells (Figure 4C), while a low MMP‐9 expression level was found in Six1‐MKD cells compared to that in Con‐MKD cells (Figure 4D). All the above findings suggest that Six1 increases expression level of MMP‐9 in macrophages.

**Figure 4:** Six1 up‐regulates matrix metalloproteinase 9 (MMP‐9) expression in macrophages. A, MMP‐9 mRNA expression level in Six1‐MOE and Vector‐M cells. B, MMP‐9 mRNA expression in Six1‐MKD and Con‐MKD cells. C, Western blotting analysis of MMP‐9 in Six1‐MOE and Vector‐M cells. D, Western blotting analysis of MMP‐9 in Six1‐MKD and Con‐MKD cells. Data are presented as means ± SD (n = 3). ***P < 0.001

### 3.5 Macrophage Six1 stimulates MMP‐9 expression and activation of STAT3‐regulated invasiveness in HA59T cells

Our findings prove that Six1 can stimulate the expression level of MMP‐9 in macrophages, but do not provide a solid connection between macrophage Six1 expression and MMP‐9 expression levels in HA59T cells. To address this, we obtained CM from Six1‐MOE, Six1‐MKD, Con‐MKD and Vector‐M macrophages, and cultured HA59T in the presence of these conditioned media for 20 minutes. As a result, MMP‐9 expression levels in HA59T cells were found to be elevated following exposure to Six1‐MOE CM compared to cells exposed to Vector‐M CM (Figure 5A). In addition, culture of HA59T cells in the presence of Six1‐MKD CM reduced MMP‐9 levels in HA59T cells compared to those in cells cultured in Con‐KD CM.

**Figure 5:** Signal transducer and activator of transcription 3 (STAT3) in HA59T cells is crucial for Six1‐induced enhanced matrix metalloproteinase 9 (MMP‐9) expression and invasion ability of HA59T cells. A, Evaluation of p‐STAT3, STAT3 and MMP‐9 expression levels in HA59T cells exposed to conditioned media (CM) from Vector‐M, Six1‐MOE, Con‐MKD and Six1‐MKD cells. B, Evaluation of P‐STAT3, STAT3 and MMP‐9 expression levels in HA59T cells exposed to the same macrophage‐derived CMs in A, with/without stattic. C and D, Quantitative analysis of HA59T cell invasion with/without stattic treatment when co‐cultured with Vector‐M or Six1‐MOE cell in the invasion assay. Data are presented as means ± SD (n = 3). *P < 0. 05

To understand the role that STAT3 activity plays in the increase of macrophage Six1‐mediated MMP‐9 expression in cancer cells, we used the STAT3 inhibitor stattic, to alter STAT3 activation levels in HA59T. After treatment with 5 μmol/L stattic for 24 hours, HA59T cells were then cultured with CM derived from Six1‐MOE or Vector‐M cells. As a result, lower MMP‐9 and phospho‐Tyr705‐STAT3 (p‐STAT3) expression levels were found in HA59T cells cultured in the presence of CM from Six1‐MOE or Vector‐M cells (Figure 5B). Nevertheless, among these two conditions, Six1‐MOE CM showed a stronger ability to reverse stattic‐triggered inhibition of MMP‐9 expression than Vector‐M CM (Figure 5B). The above findings prove the involvement of STAT3 activation in the Six1‐induced increase in MMP‐9 expression in HA59T cells.

The involvement of activated STAT3 in the invasiveness of HA59T cells stimulated by macrophage Six1 was further explored. After being treated with/without stattic, HA59T cells were evaluated for their invasiveness in the presence of Six1‐MOE or Vector‐M cells. Figure 5C and D demonstrated that stattic caused a decline number of invading HA59T cells when cultured together with Six1‐MOE or Vector‐M cells. However, compared to Vector‐M cells, Six1‐MOE cells relieved the inhibition of HA59T invasiveness caused by stattic. In summary, activation of STAT3 in HA59T cells partly accounts for the elevated invasiveness of HA59T cells induced by macrophage Six1 expression.

### 3.6 Involvement of p65 in the macrophage Six1‐stimulated MMP‐9 and IL‐6 expression

From the above findings, we assumed that macrophage Six1 can enhance the expression level of secreted factor IL‐6, which subsequently leads to STAT3 phosphorylation in HA59T cells. In agreement with this, there was a clear up‐regulation of IL‐6 mRNA expression in Six1‐MOE cells compared to that in Vector‐M cells (Figure 6A), whereas IL‐6 mRNA expression level was decreased in Six1‐MKD cells compared to that in Con‐MKD cells (Figure 6B).

**Figure 6:** p65 is involved in Six1‐mediated up‐regulation of IL‐6 and matrix metalloproteinase 9 (MMP‐9) in macrophages. A, IL‐6 mRNA expression levels in Six1‐MOE and Vector‐M cells were detected by real‐time RT‐PCR. B, IL‐6 mRNA expression levels in Six1‐MKD and Con‐MKD cells. C, The effect of Six1 on p65 expression in macrophages. D, Efficiency of simultaneous transfection of siRNA and plasmids was assessed by western blotting. E, Relative mRNA expression levels of Six1, IL‐6 and MMP‐9 in Vector‐M + NC and Vector‐M + p65i cells. F, Six1, IL‐6 and MMP‐9 relative mRNA expression levels in Six1‐MOE + NC and Six1‐MOE + p65i cells. G, IL‐6 level was analysed by ELISA. H, Mode of macrophage Six1 regulating HCC cells invasion. Data are presented as means ± SD (n = 3). *P < 0.05; **P < 0.01

It is widely known that macrophage IL‐6, being a major target gene for p65, can cause tumour growth, which made us wonder if p65 was also involved in the Six1‐mediated induction of IL‐6 expression in macrophages.^24^, ^25^ To address this, we initially examined the influence of macrophage Six1 expression on p65 protein expression. Compared to Vector‐M cells, p65 protein levels were clearly increased in Six1 overexpressing macrophages (Six1‐MOE cells), whereas p65 expression was decreased in Six1‐MKD cells (Figure 6C). To further explore the effect of p65 on macrophage Six1‐stimulated IL‐6 expression, we knocked down p65 with siRNA. Macrophages were co‐transfected with either pCMV‐XL4 Six1 (Six1‐MOE) or Vector‐M plasmid DNAs, and either a siRNA targeting p65 (p65i) or a control siRNA (NC), after which p65 and Six1 expression levels were assessed by western blotting (Figure 6D). Six1 mRNA levels were evaluated in cells transfected with the following plasmid/siRNA combinations, Vector‐M + NC, Vector‐M + p65i, Six1‐MOE + NC and Six1‐MOE + p65i (Figure 6E**)**. Nevertheless, Six1‐induced IL‐6 overexpression was abolished by the p65 siRNA in Six1‐MOE + p65i transfected cells (Figure 6F). The IL‐6 mRNA expression in Six1‐MOE + p65i transfected cells was much higher than in Six1‐MOE + p65i transfected cells. These data therefore establish that p65 mediates Six1‐induction of IL‐6 expression in macrophages. Subsequently, we explored whether p65 was also involved in Six1‐stimulated MMP‐9 expression in macrophages. These data showed that MMP‐9 levels in Six1‐MOE + p65i transfected cells were not markedly lower than they were in Six1‐MOE + NC transfected cells. However, the p65 siRNA significantly impeded the elevation of MMP‐9 expression mediated by macrophage Six1 expression (Figure 6F and G). These data indicate that there is a regulatory role for p65 in Six1‐induced MMP‐9 expression in macrophages.

## 4 DISCUSSION

Previous research has shown that up‐regulation of Six1 in HCC is associated with a worse tumour grade.^26^ Using a multivariate analysis, it has also been suggested that Six1 could be an independent risk factor for tumour recurrence, therefore having a significant negative impact on survivability.^16^, ^27^ Additionally, compared to those in HCC patients without metastases, Six1 expression levels were high in tissues from patients with metastases.^28^ All these data provide persuasive evidence to prove the ability of Six1 to facilitate progression and metastasis in HCC (Figure 6H).

Currently, studies examining the impact of Six1 on tumour progression have primarily involved various kinds of cancer cells.^29^, ^30^ Our study showed that there was significantly more Six1 expression in TAMs in HCC tissues than in neighbouring non‐tumour tissues. Because of the close relationship, high Six1 expression and tumour metastasis and invasion,^30^ we hypothesized that the expression of Six1 in macrophages may contribute to promoting the invasive process in tumour cells. The human monocyte cell line THP‐1 is a well‐known model, suitable for studying the regulatory role of monocytes as well as macrophages.^31^, ^32^ Here, we used THP‐1 cells to explore how Six1 expression in macrophages might affect tumour invasion. We successfully demonstrated that overexpression of Six1 in macrophages stimulates HA59T cell invasiveness by increasing MMP‐9 levels in both HA59T tumour cells and macrophages. Activated STAT3 appeared to modulate Six1 expression, up‐regulate MMP‐9 and improve the invasive ability of HA59T cells.

MMP‐9 is one example of several proteolytic enzymes that can decrease extracellular matrix and is indispensable for invasiveness, thereby promoting cancerous invasion of nearby tissues.^33^, ^34^ It has been shown that MMP‐9 is closely related to lymphatic metastasis and unfavourable prognosis in laryngeal cancer.^35^ In our current research, the relationship between increased Six1 expression in HCC samples and the elevation MMP‐9 expression was explored. Being produced from both tumour and stroma cells, particularly macrophages, MMP‐9 is known to have a central position in cancer metastasis, invasion and angiogenesis. Our studies suggest that Six1 in macrophage can increase MMP‐9 expression level in both HA59T cells and macrophages.

In the malignant transition, increased STAT3 tyrosine phosphorylation (p‐STAT3) is observed in around 70% of haematological malignancies or solid tumours.^36^ Increased p‐STAT3 levels are involved in both enhanced metastasis and invasion in different types of cancers.^36^, ^37^ Accumulating evidence suggests that activated STAT3 is intimately connected with MMP‐9 expression levels and extracellular matrix remodelling, which increases the invasiveness of cancer cells, especially cancers that have developed drug resistance.^38^, ^39^ Our research has demonstrated that STAT3 activation is as least partly responsible for the up‐regulation of MMP‐9 level in HA59T cells induced by macrophage Six1 expression. We propose that this novel STAT3‐MMP‐9 pathway is associated with the Six1‐triggered invasion of cancer cells.

Based on innumerable studies, TAMs are believed to relate to elevated rates of metastasis and angiogenesis by activating different growth and cell factors. NF‐κB has proven to be a significant factor in regulating genetic transcription inside macrophages and its activation has been demonstrated to enhance carcinogenesis in some cancers, particularly those related to inflammation.^40^ A gene chip expression profile analysis revealed that overexpression of Six1 could cause an elevation of certain NF‐κB downstream target gene IL‐6.^41^ In another study, the down‐regulation of Six1 was found to be able to deactivate NF‐κB and decrease MMP‐9 levels.^42^ Aligned with these previous findings, our study revealed that Six1 is a necessary element for activating p65 in macrophages. Our study highlighted the importance of the role of p65 in the Six1‐triggered increases in MMP‐9 and IL‐6 expression levels in macrophages. The co‐cultivation of cancer cells with macrophages suggested that different secreted factors, such as IL‐6, derived from activated macrophages could activate STAT3 in the cancer cells. Activation of STAT3 in cancer cells mediates the macrophage effect on the tumour cell. Our study revealed that macrophage Six1 expression increased IL‐6 expression, which then led to the activation of STAT3 in cancer cells. Nevertheless, the contribution of Six1 to tumour development could be related to many other cell and growth factors, and more researches are required to identify the exact mechanism by which Six1 in macrophages impacts the function of IL‐6, or other cell growth factors involved in cancer cell metastasis.

A previous study established the existence of two constitutive groups of macrophages: M1 and M2 macrophages.^43^, ^44^ In several tumours examined, TAMs resemble M2 macrophages.^45^ This kind of classification has certain limitations in that it may not be applicable in the sophisticated tumour microenvironment.^45^, ^46^ Moreover, recent gene expression profiling studies have identified the macrophages in the tumour microenvironment as being either M1 or M2.^47^ Apart from TNF‐α, another inflammatory cytokine IL‐6, the up‐regulation of which was induced by overexpression of Six1, also nurtures an inflammatory environment, thus leading to chronic colitis and even colon cancer.

Overall, increased Six1 expression was detected in the TAMs in HCC. Macrophage Six1 was found to be able to stimulate HA59T cell invasion by up‐regulating IL‐6 and MMP‐9 expression via p65. Six1‐MOE‐conditioned media triggers the activation of STAT3, which then leads to an increase in MMP‐9 expression and an elevated invasive ability in HA59T cells. This research has shown the importance of Six1 in macrophages in terms of facilitating invasion in HCC and cell metastases, thus suggesting a new direction for the development of novel therapeutics to treat HCC.

## CONFLICT OF INTEREST

The authors declare no conflict of interest.

## AUTHOR CONTRIBUTIONS

In this work, Yongyu Zhang and Ming Xiu conceived the study and designed the experiments. Shiji Wang and Zhongmin Liu contributed to the data collection; Lewei Yang and Jian Liu performed the data analysis and interpreted the results. Yongyu Zhang wrote the manuscript; Ming Xiu contributed to the critical revision of article. All authors read and approved the final manuscript.
